The article "Effects of Daily Activities and Position on Kinematics and Contact Mechanics of Dual Mobility Hip Implant" was published in 2020. Journal: J Healthc Eng.

# Effects of Daily Activities and Position on Kinematics and Contact Mechanics of Dual Mobility Hip Implant

**DOI:** 10.1155/2020/8103523

**Published:** 2020-03-14

**Authors:** Yongchang Gao, Xin Zhao, Shibin Chen, Jing Zhang, Zhenxian Chen, Zhongmin Jin

**Affiliations:** ^1^National Engineering Laboratory for Highway Maintenance Equipment, Chang'an University, 710064 Xi'an, Shaanxi, China; ^2^State Key Laboratory for Manufacturing System Engineering, School of Mechanical Engineering, Xi'an Jiaotong University, 710049 Xi'an, Shaanxi, China; ^3^Institute of Medical and Biological Engineering, School of Mechanical Engineering, University of Leeds, Leeds LS2 9JT, UK

## Abstract

Dual mobility hip implants have been widely introduced to overcome dislocation in recent years. However, the potential influence of different gaits on kinematics and contact mechanics for dual mobility hip implants is still unclear. Furthermore, a large range of motion coupling with the implant position, especially high inclination or anteversion angle, may result in poor kinematics and contact mechanics. A previously developed dynamic finite element method was adopted in this study to examine the kinematics and corresponding stability of dual mobility hip implants under different gaits coupling with different inclinations or anteversion angles. The results showed only inner relative sliding under knee-bending for dual mobility hip implants under moderate inclination and anteversion angles, whereas an anteversion angle of 25° induced both impingement and consequent relative sliding of the outer articulation. However, the impingement (between the stem neck and the liner inner rim) indeed happened under stair-climbing and sitting-down/stand-up as well as combined movements when inclination and anteversion angles were set as 45° and 0°, respectively, and this finally led to relative sliding at the outer articulation. A high inclination angle did not worsen both the impingement and related outer sliding compared to modest inclination and anteversion angles of the liner, but a high anteversion angle prolonged the period of both the impingement and the outer relative sliding. The extreme motions and high anteversion angles are hardly inevitable, and they indeed lead to motions at both articulations for dual mobility hip implants.

## 1. Introduction

Dual mobility hip implants have been introduced extensively to prevent long-term dislocation of artificial hip joints [1, 2]. After decades of trials in clinics, this kind of prosthesis has shown excellent stability and lesser dislocation rate compared to conventional hip implants, especially for the conditions with a high risk of dislocation such as revisions and acetabular bone defect [2–4]. Therefore, dual mobility hip implants are considered to be the most efficient way to guard against dislocation of artificial hip joints after surgery. Till now, this type of implant has been widely used around the world, particularly in Europe [5, 6].

The article "Effects of Daily Activities and Position on Kinematics and Contact Mechanics of Dual Mobility Hip Implant" was published in 2020. Journal: J Healthc Eng.

The dual mobility hip implant is mainly composed of a back shell, an intermediate liner, and a modular femoral head (a stem is coupled). Because the liner is not constrained onto the back shell anymore as the conventional hip joint done, it is intended to be mobile and thus two articulations are introduced (inner articulation: femoral head and the inner surface of the liner; outer articulation: inner surface of the back shell and the outer surface of the back shell) for this kind of implant. The liner will remain static when the stem rotates during walking movement, and thus, only inner articulation relative motion occurs if both articulations are of similar lubrication. However, it is possible that the stem neck impinges the inner rim of the liner when high anteversion angle is initially set for the liner and finally leads to rotation of the liner together with the stem (relative motion at the outer articulation) under the same walking activity. Both of these two different relative motions during walking gait cycle were observed in the studies by Gao et al. [7, 8]. Besides high anteversion angle of the liner, large range of motions like climbing/descending stairs and chair sitting-down/standing-up will probably result in impingement and then cause relative motion at outer articulation for the dual mobility hip implant. Thus, the dual mobility hip implant could keep excellent stability and prevent dislocation. Nevertheless, potential relative motions at both the inner and the outer articulations may lead to increased wear and consequently wear-induced osteolysis. Clinically, Geringer et al. [9] measured the wear volume of the retrieved liners of 12 dual mobility hip implants, with 10 samples examined for both the inner and outer surfaces. Adam et al. [10] also reported similar results of retrieved dual mobility hip implants. Theoretically, Fabry et al. [11] investigated the dynamic behaviour of a dual mobility hip implant under different movements and found dual motions at both the inner and the outer articulations under stair-climbing and chair down/up (the outer motion caused by impingement between the stem neck and the inner rim of the liner). These studies confirmed that a complex motion may be experienced for the dual mobility hip implant. However, the current research still does not reveal the complex biomechanics of dual mobility hip implants under different movements especially for those activities that would potentially cause impingement and consequent dual motions. Although high inclination angles have not been found to increase the wear volume of dual mobility hip implants [12, 13], it is probable that high inclination or anteversion angles would be more likely to lead to edge loading and edge wear for dual mobility hip implants, similar to conventional hip implants [14]. A previous study showed that impingement and the corresponding relative sliding of the outer articulation of the liner did not occur even at a high inclination angle of 70° under walking; however, this was not true for an anteversion angle of the liner exceeding 20° [8]. Furthermore, once a large range of movements combined with high inclination or anteversion angles of the liner would further lead to the worsening of the biomechanics of the dual mobility hip implant. This may finally worsen the stability or range of motion (ROM) for dual mobility hip implants. However, both the kinematics and stability of the dual mobility hip implant under these extreme conditions are still unclear. Therefore, this study aimed to investigate the effects of daily activities and inclination/anteversion on both the kinematics and the contact mechanics of dual mobility hip implants using a previously developed explicit dynamic finite element method.

The article "Effects of Daily Activities and Position on Kinematics and Contact Mechanics of Dual Mobility Hip Implant" was published in 2020. Journal: J Healthc Eng.

## 2. Materials and Methods

A dual mobility hip implant, including the back shell, the liner, the femoral head, and stem, was modeled as in Figure 1(a) without considering pelvis (the pelvis would not apparently affect the kinematics and contact mechanics of the prothesis). The geometry of this implant was mainly taken from Serf's dual mobility hip implant [15] including both shapes and key dimensions of all three components. The femoral head was cobalt-chromium alloy and of a diameter of 28 mm. The liner was ultra-high-molecular-weight polyethylene (UHMWPE), and its inner and outer diameters were 28.3 mm and 48.95 mm, respectively. The detailed dimensions and materials of the dual mobility hip implant are shown in Table 1. The femoral head and the stem were simplified as a fully bonded together with different material properties. According to ideal position in THR surgery, both the back shell and the liner were set at 45° inclination and 0° anteversion angles, respectively, and the femoral head originally was located at standing position (Figure 1(a)). A coordinate system was established with the origin at the center of the femoral head as in Figure 1(a); the positive *X*-axis was pointed medial, the *Z*-axis was along superior, and the *Y*-axis was perpendicular to both the *X*-axis and the *Z*-axis and towards to posterior.

The article "Effects of Daily Activities and Position on Kinematics and Contact Mechanics of Dual Mobility Hip Implant" was published in 2020. Journal: J Healthc Eng.

The dual mobility hip implant would experience different range of motions under different daily activities such as walking and knee-bending. In this study, knee-bending, stair-climbing, sitting-down/up, and combination of them were considered. The original data of these movements were from Bergmann et al. [16], and then they were slightly revised by Fabry et al. [17] (Figure 2) to generate combined movements. According to the testing of Bergmann et al., the gaits data was average value through measured patients. The motion of any activity is combined actions of flexion-extension (FE), abduction-adduction (AA), and internal-external rotation (IER). Finally, these movements were transformed into continuous incremental rotation vectors using a previously developed dynamic finite element method [18] to perform dynamic FE analysis.

Although the dual mobility hip implant is generally implanted with appropriate inclination and anteversion angles as the conventional artificial hip joint, the liner is hard to be fixed and keep the position unchanged. The ideal position of the liner in THR surgery is of 0° and 45° for inclination and anteversion angles, respectively. For other positions, the liner may be of high inclination or/and anteversion angles. These possible positions of the liner were designed to three different cases in this study. Case 1 specified the inclination angle and anteversion angle of the liner of 45° and 0° for all gaits, respectively. In Case 2, the inclination angle of 70° and anteversion angle of 0° were used for the liner, with a reference to a previous study [8]. For Case 3, the inclination angle and anteversion angles of the liner were set as 45° and 25°, respectively.

An explicit dynamic finite element method, which was developed in a previous study [18], was used to perform the biomechanical analysis, using the commercial finite element software ABAQUS 6.13 version. The FE model is shown in Figure 3(b) with the same coordinate system established as the CAD model. The back shell, the liner, the femoral head, and potential contact area of the stem were meshed by eight-node structured hexahedron elements with the element size of 0.4 mm, 1.2 mm, and 0.4 mm, respectively. The remaining portions of the stem were meshed by the four-node tetrahedron elements (the element size was about 2.5 mm). A mesh sensitivity study of the liner (important component of the dual mobility hip implant) was carried out and an appropriate element size of 1.2 mm was determined (maximum error less than 6%). The elastic modules, the Poisson ratio, and density of all parts are also listed in Table 1. The UHMWPE was treated as a nonlinear material with the yield stress of 23.56 MPa [7, 18], and it was also considered as elastic-plastic. Because the elastic moduli of both the titanium alloy and cobalt-chromium alloy were two orders of magnitude higher than those of the UHMWPE, these metallic parts were regarded as rigid-body.

The article "Effects of Daily Activities and Position on Kinematics and Contact Mechanics of Dual Mobility Hip Implant" was published in 2020. Journal: J Healthc Eng.

All three surface-to-surface contact pairs were modeled, including the back shell and liner, the liner and the femoral head, and the liner inner rim and the stem neck as shown in Figure 3(c), respectively. The prosthesis was lubricated by synovial fluid; thus friction coefficient of all contact pairs was set to be 0.08 according to the study by Banchet el al. [19]. The outer surface of the back shell was fully constrained. Both the dynamic movements and the spatial forces of different gaits introduced in Figure 2 were applied at the center of the femoral head. Then the femoral head and stem gradually rotated according to the input movement curve until the end of a gait cycle. Finally, the accumulated sliding distance and contact pressure of the inner and outer surfaces as well as the inner rim of the liner were obtained to evaluate both the kinematics and the contact mechanics of the dual mobility hip implant.

## 3. Results

The contours of the maximum accumulated sliding distances of the inner and outer surfaces of the liner at three different inclination and anteversion angles for an entire knee-bending gait cycle are shown in Figure 3. For both Case 1 and Case 2, the liner inner and outer contact areas were slightly different but the related maximum accumulated distance showed little difference during the whole knee-bending gait cycle (the liner inner and outer maximum accumulated sliding distance were about 26.5 mm and 0.7 mm, respectively). At the same time, the impingement of the liner inner rim did not occur and the related accumulated sliding distance was kept zero during the whole gait cycle for these two cases. However, the impingement between the liner inner rim and the stem neck indeed occurred for Case 3, and this led to increasing of the liner outer accumulated sliding distance but decreasing of the liner inner accumulated sliding distance. The variations of the maximum accumulated sliding distance of the liner inner and outer surfaces during the whole knee-bending gait are shown in Figure 4 for all three inclinations and anteversion cases. It can be seen that the impingement lasted from about 17% to 47.5% of the gait cycle for case 3. During the impingement period, both the accumulated sliding distance of the liner inner rim and the liner outer surface gradually increased and finally reached the maximum value of 3.8 mm and 11.9 mm, respectively. However, the maximum accumulated sliding distance of the liner inner surface was only about 19.4 mm. The results again revealed that the impingement between the stem neck and the liner inner rim did not happen and only the inner articulation experienced relative rotation for both case 1 and case 2 during the knee-bending gait cycle. Meanwhile, the contours of the maximum contact pressure of the inner and outer surfaces of the liner at three different inclination and anteversion angles for an entire knee-bending gait cycle are shown in Figure 5. The contact zone changed when the liner was set different inclinations or anteversion angles during the knee-bending movement especially for case 2, but the maximum contact pressure showed little difference among the three different cases with the values of 12.4 MPa, 3.5 MPa, and 69.2 MPa at the liner inner surface, liner outer surface, and the liner inner rim, respectively. Although the impingement between the liner inner rim and the stem neck lasted very short during the whole gait cycle, the resulted contact pressure of the liner rim was much higher than that of the liner inner and outer surfaces. The variations of the maximum contact pressure of the liner inner and outer surfaces during the whole knee-bending gait are shown in Figure 6 for different inclination and anteversion cases. For all three cases, the liner inner and outer maximum contact pressure varied with the applied forces during the whole knee-bending gait cycle. The results further revealed the time when the impingement occured under large anteversion angle of the liner and its effects on contact pressure. The maximum contact pressure of the liner inner and outer surfaces for case 1 and case 2 varied with the applied forces and overall showed little difference during most time of the gait cycle. The impingement between the liner inner rim and the stem neck happened for case 3 and lasted about 30% of the whole gait cycle. The resulted maximum contact pressure of the liner inner rim was rather high and nearly reached 70 MPa. This also resulted in both the liner inner and outer maximum contact pressure slight decreased during the impingement period but increased after the impingement comparing to the other two inclinations and anteversion cases. When it refers to ROM of the dual mobility hip implant, it seemed there was nearly no difference for three different cases (case 1: 52.1°; case 2: 52.1°; case 3: 52.1°).

The article "Effects of Daily Activities and Position on Kinematics and Contact Mechanics of Dual Mobility Hip Implant" was published in 2020. Journal: J Healthc Eng.

The contours of the maximum accumulated sliding distance at the inner and outer articulations of the liner are shown in Figure 7 at three different inclination and anteversion angles during an entire sitting-down/standing-up gait cycle. Figures 7(a) and 7(c) show that the impingement of the liner inner rim occurred during this kind of gait cycle for the inclination and anteversion angles of case 1 and case 3 and eventually resulted in the relative sliding of the liner at the outer contact surfaces. However, for the inclination and anteversion angles of case 2 shown in Figure 7(b), there was nearly no impingement happening between the liner inner rim and the stem neck. The variations of the maximum accumulated sliding distance of the liner inner and outer surfaces during the whole sitting-down/standing-up gait cycle for all three inclinations and anteversion cases are shown in Figure 8. The maximum accumulated sliding distance of the liner inner at inclination and anteversion cases 1 and 3 was obviously lower than that of case 2 (case 1: 27.3 mm; case 2: 29.7 mm; case 3: 19.5 mm). But the maximum accumulated sliding distance of the liner outer at cases 1 and 3 was much higher than that of case 2 (case 1: 5.8 mm; case 2: 0.8 mm; case 3: 17.0 mm). The maximum accumulated sliding distance of the liner inner rim was much lower than that of the liner inner and outer surfaces for both three inclination and anteversion angles (case 1: 1.0 mm; case 2: 0.1 mm; case 3: 3.9 mm). However, the impingement period only occupied a small proportion during the whole gait cycle even under case 3 (about 22% of the gait cycle). Beyond the impingement process, only inner relative sliding occurred and the liner inner maximum accumulated sliding distance gradually increased. The ROM of the dual mobility hip implant under this activity: it seemed there was nearly no difference for three different cases (case 1: 59.0°; case 2: 59.5°; case 3: 59.0°).

The liner inner rim also experienced impingements during both stair-climbing and combined gait cycles. These impingements showed similar influence on the liner inner and outer surface maximum accumulated sliding as the sitting-downing/standing-up gait cycle; the detailed results are listed in Table 2. During the stair-climbing process, the impingement of the liner inner rim also sustained a short period in this gait cycle (the maximum value was about 16.3% under case 3). The liner inner relative sliding dominated in this gait and the corresponding maximum value (case 1: 52.3 mm; case 2: 52.6 mm; case 3: 41.1 mm) was much higher than that of the liner outer and inner rim. The accumulated sliding distance of the liner inner rim was small but apparently different for three inclination and anteversion angles (case 1: 0.2 mm; case 2: 2.2 mm; case 3: 3.9 mm), and the consequent maximum accumulated sliding distance of the liner outer surface (case 1: 4.0 mm; case 2: 3.5 mm; case 3: 16.8 mm) also showed difference. For the combined gait cycle, the lasting time of the liner inner rim impingement was less than 4% of the gait cycle (the maximum value was 3.8% of case 3). Similarly, the liner inner relative sliding dominated again and caused maximum accumulated sliding distance to be the highest (case 1: 95.6 mm; case 2: 98.6 mm; case 3: 81.8 mm). The maximum accumulated sliding distance of the liner inner rim (case 1: 0.8 mm; case 2: 2.3 mm; case 3: 3.6 mm) was very small and the caused maximum accumulated sliding distance of the liner outer surface (case 1: 4.6 mm; case 2: 4.0 mm; case 3: 16.3 mm) was a bit higher than itself. The maximum contact pressure of the liner inner and outer surfaces as well as liner inner rim under sitting-down/up, stair-climbing, and combined movements are also shown in Table 2. The ROM of the dual mobility hip implant under each of these activities also showed little difference under three different positions (shown in Table 2). Similarly, although impingement occurred and lasted very short during these movements, the resulted maximum contact pressure of the liner inner rim was extremely high.

The article "Effects of Daily Activities and Position on Kinematics and Contact Mechanics of Dual Mobility Hip Implant" was published in 2020. Journal: J Healthc Eng.

## 4. Discussion

The dual mobility hip implant may experience impingement and consequent relative sliding at both inner and outer articulations under extreme movements such as stair-climbing. However, the kinematics and the contact mechanics of dual mobility hip implants under the condition of impingement are still unclear. If the liner is at a high anteversion angle which has been proven to result in impingement between its inner rim and the stem neck in a previous study [8], this impingement may become worsen under an extreme range of motion. Therefore, the current study used a previous developed dynamic explicit finite element method to investigate the effect of both different movements and positions on kinematics and contact mechanics of dual mobility hip implants. This study predicted both contact pressure and relative sliding of the liner inner, liner inner rim, and outer surfaces under different movements and inclination/anteversion angle for dual mobility hip implants, and the accumulated sliding distance and contact pressure were output to show the effect of movements and inclination/anteversion angle on kinematics and contact mechanics of dual mobility hip implants.

Both contact pressure and the accumulated sliding distance and ROM of dual mobility hip implant under different daily activities were predicted. The main findings of this study can be concluded as three points. First, the impingement between the stem neck and the inner rim of the line occurred during sitting-down/standing-up, stairs-climbing, and combined movements. Just the impingement led to the liner rotated together with the stem and finally resulted in relative motion at the outer articulation for the dual mobility hip implant. However, the impingement did not increase the contact pressure of both inner and outer surfaces of the UHMWPE liner. Secondly, if the liner was initially set high anteversion angle, it would prolong the period of both impingement and increased consequent relative sliding distance of the outer articulation for the dual mobility hip implant. Similarly, this still did not obviously worsen the contact mechanics of the liner. Third, the dual mobility hip indeed experienced large ROM under knee-bending, sitting-down/standing-up, stairs-climbing, and combined movements. The lasting period of impingement did not obviously influence the ROM for dual mobility hip implant under these different activities.

The article "Effects of Daily Activities and Position on Kinematics and Contact Mechanics of Dual Mobility Hip Implant" was published in 2020. Journal: J Healthc Eng.

The study of Fabry et al. [11] showed that the liner of the dual mobility hip implant rotated from its initial position to a new position after one hundred gait cycles under knee-bending, sitting-down/standing-up, stairs-climbing, and combined movements, thus the inclination angle of the liner also changed during these daily activities. During this study, the rotation of the liner resulted from the impingement between the liner inner rim and the stem neck because both articulations were well lubricated (this lubrication condition would not lead to the rotation of the liner for dual mobility hip implant according to Rowe et al.'s study [20]). The current study also showed that the dual mobility hip implant experienced impingement of the liner and consequent outer articulation relative movement under sitting-down/standing-up, stairs-climbing, and combined movements. Therefore, the current study again indicated that the large range of motions of patients would result in impingement of the liner and finally lead to both inner and outer articulations relative rotations for dual mobility hip implant. However, the predicted relative movement of the liner by this study during knee-bending gait cycle was different from the result by Fabry et al. The current study showed that both the impingement of the liner and consequent outer articulation relative rotation did not occur for the dual mobility hip implant under knee-bending gait cycle if the anteversion angle was kept as zero degree (even the inclination angle reached 70 degrees), whereas they happened in Fabry et al.'s study. However, the impingement indeed happened in this gait cycle and this finally led to the liner outer relative sliding when the anteversion angle of the liner was set to be 25°. For those movements resulting in impingement of the liner of the dual mobility hip implant, the current study indicates that the inner articulation relative rotation dominated but the relative rotation of the outer articulation only occupied a small portions during one whole gait cycle. Thus, although the impingement of the liner of the dual mobility hip implant indeed occurred during large range of motions, the dual mobility still kept stability during these movements. The key benefit of this study is that the detailed impingement of the liner of the dual mobility hip implant was verified for different patients' daily activities. In addition, the quantitative values of the sliding distance at all contact zones were obtained in this study under different patients' daily activities.

The article "Effects of Daily Activities and Position on Kinematics and Contact Mechanics of Dual Mobility Hip Implant" was published in 2020. Journal: J Healthc Eng.

The dual mobility hip implant would also experience impingement of the liner under extreme anteversion angle during walking movement according to previous study [8]. The current study also reveals that the impingement of the liner would intensify when the liner was set higher anteversion angle under sitting-down/standing-up, stairs-climbing, and combined movements. Then both the relative sliding of the outer articulation and the corresponding maximum accumulated sliding distance increased because of the increasing of this impingement. Although high anteversion angle of the liner made the impingement of the liner worse, the liner still did not dislocated from the back shell. In addition, higher inclination angle (up to 70°) combining nonanteversion angle did not enhance the impingement of the liner for all kinds of patient's daily activities. It even made the liner avoid impinging the stem neck under the sitting-down/standing-up gait cycle. But the impingement indeed occurred under this gait cycle for other inclination and anteversion angles (case 1 and case 3). This may mean the dual mobility could keep excellent stability even at poor orientation of the liner and large range of patients' movements. The orientation of the liner of a dual mobility hip implant is hard to keep at a static position because of the dual mobility property of this kind of prothesis, and as a result, the liner probably could not stay at a standard orientation (45° inclination angle and 0° anteversion angle) as the conventional hip implant. A large range of motions of the dual mobility hip implant is also inevitable because of demands of daily activities of patients. Therefore, the conditions of this study that the liner was of different inclinations or anteversion angles under different daily activities may be more close to the in vivo situation. According to the results of this study, although the dual rotations of the dual mobility hip implants caused by impingement of the liner under large range of motions and high anteversion angle were inescapable for dual mobility hip implant, this did not lead to dislocation of the femoral head under these extreme conditions. This rather benefits those who under total hip replacement use the dual mobility hip implant to prevent dislocation of the implant.

The article "Effects of Daily Activities and Position on Kinematics and Contact Mechanics of Dual Mobility Hip Implant" was published in 2020. Journal: J Healthc Eng.

When it refers to contact pressure at all contact pairs during different inclinations and anteversion angles for daily activities, the impingement between the stem neck and the liner inner rim resulted in very high contact pressure at liner inner rim during the impinging period which could be harmful for the liner. However, this impingement did not apparently influence the contact pressure of both the liner inner and outer surfaces. For all daily activities, the relative motion of the inner articulation dominated for the dual mobility hip implant even under the worst position that the liner was of high anteversion angle. This probably finally led to the inner wear dominating for the dual mobility hip under extreme range of motions such as sitting-down/up and stair-climbing. This was in agreement with the result of the study by Imbert et al. [21] that the inner wear was overall much higher than the outer wear of the UHMWPE liner examined from retrieved dual mobility implants.

The current study predicted the kinematics and the contact mechanics of the dual mobility hip implant under daily activities of patients and high inclination or anteversion angle. However, several limitations should be pointed out. First, the relative experiments were still unavailable to be performed in this study. Second, the impingement and consequent relative sliding of the outer articulation for the dual mobility hip are dependent with the geometry and the size of the liner; however, only one kind of liner and constant size of liner were investigated in this study, and other geometry and sizes of the liner should be considered in the future. Third, average gaits data was used in this study; it is still needed to investigate kinematics and contact mechanics of dual mobility hip implant for a specified-patient according to his or her gait data. Besides, the soft tissue still has not been included in the FE model of the dual mobility hip implant; however, this may result in insert blocking and introprosthetic dislocation, and this should also be considered in future study.

## 5. Conclusion

Different daily activities and implant positions were considered to investigate their effects on the kinematics and the contact mechanics of a dual mobility hip implant using previous developed dynamic explicit finite element method. The impingement of the liner and consequent dual relative rotations were obtained during the movements of sitting-downing/standing-up, stairs-climbing, and their combinations even at appropriate inclination and anteversion angles of the liner (45° and 0°, respectively). When a higher inclination or anteversion angle was set for the liner, both the impingement and the outer articulation relative sliding would increase for the dual mobility hip implant. However, both the impingement and the outer articulation relative sliding did not occur during a knee-bending gait cycle even at high inclination or anteversion angles. The dual mobility hip implant indeed experienced impingement and related rotation of the liner during an increased range of motions, particularly combined with high anteversion angles. The impingement and consequent relative sliding of outer articulation for dual mobility hip implant could be inevitable because of patients' daily activities and uncertainly of the liner orientation in vivo for the dual mobility hip implant, but the inner articulation would probably dominate in both the relative motion and wear for the dual mobility hip implant under these extreme conditions.

The article "Effects of Daily Activities and Position on Kinematics and Contact Mechanics of Dual Mobility Hip Implant" was published in 2020. Journal: J Healthc Eng.

## Figures and Tables

**Figure 1:** CAD model (a) and FE model (b) as well as contact pairs (c) of the dual mobility hip implant.

**Figure 2:** Original movements data from Fabry et al. [17].

**Figure 3:** Contours of the liner (a) inner, (b) outer, and (c) inner rim maximum accumulated sliding distance (mm) under three different inclination and anteversion cases during knee-bending gait cycle.

**Figure 4:** Liner inner (a), outer (b), and inner rim (c) maximum accumulated sliding distance as a function of knee-bending gait cycle under three different inclination and anteversion angles for the dual mobility hip implant.

**Figure 5:** Contours of the liner (a) inner, (b) outer, and (c) inner rim maximum contact pressure (MPa) under three different inclination and anteversion cases during knee-bending gait cycle.

**Figure 6:** Liner inner (a), outer (b), and inner rim (c) maximum contact pressure as a function of knee-bending gait cycle under three different inclination and anteversion angles for the dual mobility hip implant.

**Figure 7:** Contours of the liner (a) inner, (b) outer, and (c) inner rim maximum accumulated sliding distance (mm) under three different inclination and anteversion cases during sitting-down/standing-up gait cycle.

**Figure 8:** Liner inner (a), outer (b), and inner rim (c) maximum accumulated sliding distance as a function of sitting-down/standing-up gait cycle under three different inclination and anteversion angles for the dual mobility hip implant.

The article "Effects of Daily Activities and Position on Kinematics and Contact Mechanics of Dual Mobility Hip Implant" was published in 2020. Journal: J Healthc Eng.

**Table 1:** Key geometry and material parameters of dual mobility hip implant.

	Inner radius (mm)	Outer radius (mm)	Materials	Density (g/mm^3)^	Elastic modulus (GPa)	Poisson's ratio
Femoral head	—	14.000	CoCr alloy	7.61	217	0.30
Liner	14.150	24.475	UHMWPE	0.93	1	0.45
Stem	—	—	Ti alloy	4.4	110	0.3
Back shell	24.500	27.500	CoCr alloy	7.61	217	0.30

**Table 2:** Dual motions of the dual mobility hip implant under large range of patient's activities.

	Inclination and anteversion angles	Impingement		Maximum accumulated sliding distance (mm)	Maximum contact pressure (MPa)	Range of motion (degree)
		Occur	Sustain period during whole gait cycle	Inner/outer/inner rim	Inner/outer/inner rim	
Sitting-down/up	Case 1	Yes	22.5∼27.5	27.3/5.8/1.0	12.6/4.1/50.5	59.0
	Case 2	No	0	29.7/0/0	13.3/4.1/0	59.5
	Case 3	Yes	7.5∼25	19.5/17.0/3.9	12.5/3.9/73.4	59.0

Upstairs	Case 1	Yes	66.3∼69.3	52.3/4./0.2	13.6/4.6/41.9	65.3
	Case 2	Yes	63.8∼66.7	25.6/3.5/2.2	13.5/4.7/50.5	57.3
	Case 3	Yes	6.3∼21.3, 63.8∼66.8	41.1/16.8/3.9	15.0/4.8/57.8	57.3

Combined gait	Case 1	Yes	6.5∼6.7	95.6/4.6/0.8	14.4/4.6/48.6	71.1
	Case 2	Yes	57.0∼61.0	98.6/4.0/2.3	13.2/4.4/38.9	70.5
	Case 3	Yes	3.1∼6.4	81.8/16.3/3.6	14.1/4.8/98.2	71.1

Knee-bending	Case 1	No	0	95.6/0/0	14.4/4.6/48.6	52.1
	Case 2	No	0	98.6/0/0	13.2/4.4/38.9	52.1
	Case 3	Yes	3.1∼6.4	81.8/16.3/3.6	14.1/4.8/98.2	52.1

## Data Availability

The data used to support the findings of this study are available from the corresponding author upon request.
